The article "Noninvasive Prototype for Type 2 Diabetes Detection" was published in 2021. Journal: J Healthc Eng.

# Noninvasive Prototype for Type 2 Diabetes Detection

**DOI:** 10.1155/2021/8077665

**Published:** 2021-11-09

**Authors:** Javier Ferney Castillo García, Jesús Hamilton Ortiz, Osamah Ibrahim Khalaf, Adrián David Valencia Hernández, Luis Carlos Rodríguez Timaná

**Affiliations:** ^1^Universidad Santiago de Cali, Facultad de Ingeniería, Cali, Colombia; ^2^MOABITER, Berlin, Germany; ^3^Al-Nahrain University, Al-Nahrain Nano Renewable Energy Research Center, Baghdad, Iraq

## Abstract

The present work demonstrates the design and implementation of a human-safe, portable, noninvasive device capable of predicting type 2 diabetes, using electrical bioimpedance and biometric features to train an artificial learning machine using an active learning algorithm based on population selection. In addition, there is an API with a graphical interface that allows the prediction and storage of data when the characteristics of the person are sent. The results obtained show an accuracy higher than 90% with statistical significance (*p* < 0.05). The Kappa coefficient values were higher than 0.9, showing that the device has a good predictive capacity which would allow the screening process of type 2 diabetes. This development contributes to preventive medicine and makes it possible to determine at a low cost, comfortably, without medical preparation, and in less than 2 minutes whether a person has type 2 diabetes.

## 1. Introduction

Diabetes is a serious chronic disease, which develops when the pancreas does not produce enough insulin (a hormone that regulates the level of glucose or sugar in the blood) or when the body cannot use this hormone effectively [1]. According to estimates by the World Health Organization, 422 million adults worldwide had diabetes in 2014, compared to 108 million by 1980 and at least 50% of people who suffer from it do not know it [1]. The WHO has also indicated that diabetes has tripled in the last 20 years. Globally, it has gone from around 151 million people with diabetes in 2000 to 463 million in early 2020. All this makes diabetes the health problem that has increased the most throughout the century [1].

The most popular methods for diagnosing diabetes such as FPG (fasting plasma glucose) and OGTT (oral glucose tolerance test) are invasive and painful methods that usually take longer than a bioimpedance measurement [2]. For the diagnosis of diabetes, the glycosylated hemoglobin (A1C) test is performed. This blood test indicates the average blood sugar level for the past two to three months. This test measures the percentage of sugar in the blood bound to the protein in red blood cells that carry hemoglobin (oxygen). The higher the blood sugar level, the greater the amount of hemoglobin with glucose. An A1C level of 6.5 percent or higher on two separate tests indicates the presence of diabetes. If a diagnosis of diabetes is received, the doctor may do a blood test to determine the presence of the autoantibodies that are common in type 1 diabetes. These tests help distinguish between type 1 diabetes and type 2 diabetes when the diagnosis is uncertain. The presence of ketone bodies (products derived from the breakdown of fat) in the urine also suggests type 1 diabetes rather than type 2 [3].

The article "Noninvasive Prototype for Type 2 Diabetes Detection" was published in 2021. Journal: J Healthc Eng.

Electrical bioimpedance represents the opposition of a biological medium to the passage of alternating current and has resistance and reactance components [4]. The resistance (*R*) is conditioned by the resistivity of the different tissues of the human body to electrical conduction. Fat and bone tissues have high resistivity, while intracellular and extracellular fluids easily conduct electrical current [5]. The reactance (*Xc*) in the biological environment is produced by the insulating effect of the cell membranes, which behave like capacitors charging and discharging the passage of current. In other words, while resistance (*R*) determines the body's hydration status, reactance (Xc) determines its nutritional status (Quesada Leyva, León Ramentol, Betancourt Bethencourt, and Nicolau Pestana [6]).

Type 2 saccharin diabetes (previously called noninsulin-dependent or adult-onset diabetes) is caused by the body not using the insulin it produces effectively. Most diabetics have type 2 (T2D), which is largely due to excess weight and lack of physical activity. The symptoms of type 2 diabetes can be like those of type 1 but are often less severe. Consequently, it is sometimes diagnosed several years after the first symptoms appear when complications have already appeared. Until recently, this type of diabetes was only seen in adults, but today it is increasingly being diagnosed in children.

Apart from bioimpedance, there are other noninvasive techniques that allow the evaluation of diabetes. Photoplethysmography is an alternative; it is just that a sensor is required for heart rhythm analysis, which can be expensive. There are also other developments given with bioimpedance but ultimately require comparisons (correlation analysis) with invasive glucose tests.

The figures and circumstances determine the importance of looking for methods that are fast, accurate, easily accessible, and in addition, low cost, which allow predicting with high probability that a person has diabetes. In the COVID-19 pandemic, people with diabetes mellitus have been one of the most vulnerable populations, since they have a greater probability of dying and having more serious conditions due to the infection, compared to the general population [3]. Diabetes is a highly prevalent disease throughout the world. It is estimated that around 415 million people currently suffer from it and that number will increase by just over 50% by 2040. It is estimated that the majority of emergency rooms will be for diabetics [7].

The article "Noninvasive Prototype for Type 2 Diabetes Detection" was published in 2021. Journal: J Healthc Eng.

Therefore, in accordance with the aforementioned, our work proposes a portable, noninvasive, and low-cost prototype capable of predicting type 2 diabetes, using electrical and biometric bioimpedance characteristics to train an artificial learning machine implementing an active learning algorithm based on population selection. The prototype implemented is detailed in the following.

## 2. Materials and Methods

### 2.1. Description of the Acquisition Prototype

The acquisition device has two main components. The first component is the PmodIA, which is an impedance analyzer built based on the AD5933 integrated circuit. The PmodIA module measures impedance values ranging from 10 [Ω] to 10 [MΩ] and uses a frequency sweep, a programmable gain amplifier, and a 13-bit temperature sensor. It uses the I2C communication protocol and has the formulas for calculating impedance and frequency settings [8]. The second component is the ESP32, which is a System on a Chip (SoC) with Wi-Fi and Bluetooth connection capabilities, a 32-bit Xtense® single-/dual-core microprocessor with a capacity of up to 600 instructions per second, a 448 KB RAM memory, 34 general-purpose pins, 18 channels of analog-digital conversion, among other functionalities [9]. This microprocessor is usually distributed on development boards with all the components it needs to function, for example, the ESP32-OLED-BAT, which has an integrated OLED screen and a battery holder. The brands Skintac and 3M were compared to choose the electrodes.  Table 1 shows the list of instruments and modules used in the development of the prototype.

The prototype is composed of the bioimpedance analyzer module, which applies and reads electric current through people's bodies. The ESP32 is used as a data processing microcontroller, which reads the signal from the previous module and saves the results to be then processed mathematically. To have a proper contact between the skin and the bioimpedance module, an appropriate means such as the electrodes must be used and finally, there are batteries to be able to make the equipment wireless and comfortable at the time of the tests.

#### 2.1.1. Configuration and Calibration of the Noninvasive Prototype

Table 2 shows the values selected for the module configuration.

The prototype delivers values with the labels real (*Rr*) and imaginary (*Ir*) for each frequency. However, these values do not correspond to the true values of the real and imaginary parts of the impedance. To obtain the correct values, the calibration must first be carried out by following these steps.

The article "Noninvasive Prototype for Type 2 Diabetes Detection" was published in 2021. Journal: J Healthc Eng.

The magnitude is calculated with (1), using the calibration resistor.

(1) $$\begin{array}{c} \mathrm{magnitude}=\;\sqrt{Rr^{2}+Ir^{2}}. \end{array}$$

Then, the FG (gain factor) is calculated, which is the gain obtained using the calibration resistance and allows calculating the impedance magnitude of the new measurements; this is calculated by

(2) $$\begin{array}{c} \text{FG}=\frac{1}{R_{\mathrm{calibration}}/\mathrm{magnitude}}\text{ .} \end{array}$$

To obtain the value of the system phase (*Z* phase), equation (3) is used with the calibration resistance.

(3) $$\begin{array}{c} \mathrm{phase}=\;\tan^{-1}\left(\frac{Ir}{Rr}\right). \end{array}$$

The FG and phase values are calculated for each one of the frequencies and used as calibration values. Therefore, for a new measurement, equation (4) is used from which the impedance values are obtained and equation (3) is used to obtain the phase of the unknown measurement; finally, with the difference between the phase of the unknown measurement and the phase of the system (phase*Z*), the calibrated phase (phase*C*) is obtained as shown in equation (5).

(4) $$\begin{array}{c} \mathrm{impedance}=\frac{1}{\mathrm{FG}*\mathrm{magnitude}}, \end{array}$$

(5) $$\begin{array}{c} \mathrm{phase}C=\mathrm{new}\;\mathrm{phase}\;\mathrm{measure}-\mathrm{phase}Z. \end{array}$$

The values of the real and imaginary parts of the calibrated impedance are obtained with equations (6) and (7).

(6) $$\begin{array}{c} \text{real}=\mathrm{impedance}*\;\cos\left(\mathrm{phase}C\right), \end{array}$$

(7) $$\begin{array}{c} \mathrm{imaginary}=\mathrm{impedance}*\;\sin\left(\mathrm{phase}C\right). \end{array}$$

To verify the calibration of the prototype, the percentage of error is calculated by

(8) $$\begin{array}{c} \mathrm{percentage}\;\mathrm{of}\;\mathrm{error}=\frac{vt-vm}{vt}*100, \end{array}$$

where *vt* is the theoretical impedance value using a 100 Ω resistor with a 100 nF capacitor in series and *vm* is the value measured using the PmodIA.

With the implementation of this mathematics, something important is assured and it is the calibration of the prototype. All electronic equipment requires handling a reference standard that allows you to obtain true and accurate results. If the previously described equations are not implemented, the prototype can deliver any result and the study would not be valid and important.

#### 2.1.2. ESP32 Programming

The ESP32 is a low energy consumption microcontroller, which due to its size turns out to be powerful for processing different tasks. This device has an integrated processor with interfaces that allows connection with various peripherals. Using FreeRTOS, which is an open-source C library, an operating system for microcontrollers is implemented. With this library, the microcontroller can execute at least two tasks in parallel or manage the execution of tasks. With this control, it is possible to make the ESP32 communicate with the PmodIA, manage the OLED screen, select from a menu using four buttons, and connect to the Wi-Fi network when necessary, making use of the task manager.

The article "Noninvasive Prototype for Type 2 Diabetes Detection" was published in 2021. Journal: J Healthc Eng.

### 2.2. API Description

An API that facilitates patient interaction with the device was developed. With this interface, the person can easily view the results indicating whether they have type 2 diabetes. The API was made in the Python programming language using the Flask, HTML, and CSS framework for the creation of the user interface. Data storage is implemented in the SQLite database, the API implementation used Amazon web services, and EC2 t2 microinstance was selected, with Ubuntu Linux/UNIX operating system with 30G of storage and a virtual core.

The API graphical interface, apart from allowing you to view and download the data sent, allows you to retrain the learning machine with the new data and download the generated model in a file with the extension (.p) to be used in Python and a file with the extension (.h) for use in microcontrollers.

### 2.3. Selection of Bioimpedance Characteristics

Rodríguez Timaná and Castillo García [10] in their work on characterizing people with T2D using bioimpedance were able to identify that people with T2D have a higher concentration of glucose, so their impedance response is different from that of healthy people since the signal must pass through more cells that contain glucose which makes them less conductive [11]. In addition, Timaná and Castillo used a 256-frequency sweep in their study. Using this number of frequencies causes a total of 1024 characteristics to be generated, which include values of magnitude, phase, real part, and imaginary part of the impedance (Rodríguez Timaná and [12]). This number of features is too high for statistical analysis of the machine learning model.

Considering the above, in this work, only 4 frequencies were used, which allows facilitating the implementation using the EPS32 and it is also possible to perform a correct and feasible statistical analysis. This process of choosing the most relevant characteristics begins with a selection of frequencies. The chosen frequencies were 4 (10000 Hz, 32400 Hz, 54800 Hz, and 77200 Hz). These frequencies are ideal to have an adequate penetration in the cells of the tissue; in addition, they allow to have a good representation of the signal and therefore good results with little demand for hardware and software.

The article "Noninvasive Prototype for Type 2 Diabetes Detection" was published in 2021. Journal: J Healthc Eng.

Figure 1 shows the information model, where it starts with the Amazon web services that store and deploy the application. Then, there is the login process which guarantees that only authorized personnel can view, add, update, and delete data. Each of the previous actions executes its process that oversees verifying, consulting, or modifying the data stored in the database.

This information model allows having an organized structure for the validation and protection of the data entered in addition to integrating the BDD prototype with the Internet of things and guaranteeing autonomous operation without the need for physical connections to computers to share data.

To obtain the best results, statistical chi-square tests are carried out that examine the differences between the observed and expected characteristics [13]. The test delivers a probabilistic value (*p* value) which, being less than 5%, means that the characteristics used are significant to obtain the expected ones. In addition, the Hosmer test is carried out, which allows examining the general fit of the model [14], and just like the chi-square, when obtaining a *p* value lower than 5%, it is established that the model is significant to predict the selected characteristic. The previous tests are used with the four selected frequencies and the biometric characteristics of age, weight, sex, and height to make up a total of 20 characteristics or attributes.

### 2.4. Machine Learning Selection

Machine learning is a subfield of artificial intelligence that simulates human intelligence processes such as learning, reasoning, and self-correction [15]. There are many types of machine learning algorithms, among which the most popular are as follows.

#### 2.4.1. Logistic Regression (LR)

It is a linear classifier and uses the logistic function to evaluate the class assigned to a prediction. The logistic function is presented as [16]

(9) $$\begin{array}{c} P=\frac{1}{1+e^{-\text{h}}}, \end{array}$$

where *P* is the prediction of the label and *h* is the point multiplication of the vector of characteristics and vector of weights plus the bias.

#### 2.4.2. Artificial Neural Network (ANN)

It is a computational model inspired by the human brain in the sense of using interconnected units called neurons, which learn by experience, usually consisting of one or more input layers, hidden layers, and output layers [17].

#### 2.4.3. K-Nearest Neighbor (KNN)

It is based on the idea of the closest patterns to the target. This classifier assigns the class label to most of the closest *K* patterns in data space [18].

The article "Noninvasive Prototype for Type 2 Diabetes Detection" was published in 2021. Journal: J Healthc Eng.

#### 2.4.4. Support Vector Machines (SVM)

These look for a linear decision surface and use values called *C* which is a parameter to control errors based on the cost margin function and gamma which is the Gaussian kernel that allows determining the variance [19].

To select the machine learning algorithm, tests were carried out with different logistic regression machines, 3-layer ANN, modifying the number of neurons to conform to different architectures, then with KN machines testing from 1 to 10 neighbors, and finally, with SVM machines with C values of 0.01, 0.03, 0.1,0.3, 1, 3, 10, and 30 and range of 0.01, 0.03, 0.1, 0.3, 1, 3, 10, and 30. In the Results section, the chosen learning machine and its correct explanation are indicated.

### 2.5. Description of the Active Training Algorithm Based on Seed Selection (ATSS)

Next, an algorithm is presented that uses a reduced number of samples for initial training, and as the samples are introduced, it updates the initial model obtained, in accordance with the increase in performance indicators.

The algorithm is based on the following concepts: Silhouette's Width (SW), which is an indicator that allows the interpretation of cohesion, which is the intraclass distance, and the separation, which is a measure of the distance between classes [12]. The measure of SW is presented as

(10) $$\begin{array}{c} S_{i}=\left\{\begin{array}{c} 1-\frac{a_{i}}{b_{i}},\;\text{if }a_{i}<b_{i}\\ 0,\text{ if }a_{i}=b_{i}\\ \frac{b_{i}}{a_{i}}-1,\text{ if }a_{i}>b_{i} \end{array}\right\}, \end{array}$$

where *a*_*i*_ is the average Euclidean distance of point *i* with respect to the samples of its same class and *b*_*i*_ is the average Euclidean distance of point *i* with respect to the samples of the other classes. For this study, the closer *S*_*i*_ is to 1, the closer it will be to the samples of its own class and the further it will be from the samples of the other classes.

Classification performance indicators are calculated with (11) to (13):

(11) $$\begin{array}{c} \mathrm{accuracy}=\frac{\text{TP}+\text{TN}}{\text{TP}+\text{TN}+\text{FP}+\text{FN}}, \end{array}$$

(12) $$\begin{array}{c} \mathrm{precision}=\frac{\text{TP}}{\text{TP}+\text{FP}}, \end{array}$$

(13) $$\begin{array}{c} \mathrm{recall}=\frac{\text{TP}}{\text{TP}+\text{FN}}, \end{array}$$

where TP is the true positives that correspond to the labels that were correctly predicted and are positive. TN is the true negatives that correspond to the labels that correspond to negative predictions. FP are false positives that correspond to the labels that were predicted negative when positive and FN are false negatives that correspond to the labels that were predicted positive when they were negative.

The article "Noninvasive Prototype for Type 2 Diabetes Detection" was published in 2021. Journal: J Healthc Eng.

The initial population or seed samples are taken with 10% of the training data that present the highest SW values. Then, the size of the final population is defined, and this value allows limiting the number of new entries to reduce the computational cost of training; if the maximum population is not reached, a new sample is added, and if it is reached, the sample with the lowest SW value will be replaced by the new sample. To accept or exchange a sample, the following conditions apply:

1. The SW value of the new sample must be greater than the lowest of the SW values of the current data
2. When training with that sample, the accuracy indicator must increase or stay the same and at least one of the other performance indicators must increase

### 2.6. Experimental Phase: Setup for Testing

To ensure that patients and users do not have adverse effects from the use of the device, which is a priority, the international standard of protocols and standards IEC 60601-1 must be considered. It presents all the testing requirements for protection from possible hazards [20] as the leakage currents that are produced by the insulation of the conductors and four parameters are defined: earth leakage current, envelope leakage current, patient leakage current, and patient auxiliary current [21].

The location of the electrodes is essential to obtain a correct bioimpedance measurement. These electrodes must be at a distance less than 4 cm between them; otherwise, there may be interferences and, therefore, erroneous values of resistance and reactance. Impedance measurements can be taken in a supine or sitting position and the electrodes must be placed on the wrist, this area being free of hair and, in addition, little exposed to the sun or other aspects that negatively affect the bioimpedance measurement. When implementing machine learning, as many variables as possible should be controlled to ensure that the classification uses the same characteristics for each sample. Factors such as sweat, hair, voluntary and involuntary muscle movements, and tickling reflexes are difficult to control in other parts of the body such as the chest, back, forehead, and sole of the foot. That is why the results could be affected by any of the variables mentioned above if the location of the electrodes was to be modified.

#### 2.6.1. Sampling and Database Creation

A database for the characterization of people was generated using the data acquisition device and the API, which together were called BDD (Bioimpedance Diabetes Detector), this database consists of 256 samples and 20 characteristics, the participating population was 53 people, including 34 women and 19 men, and the age range was between 19 and 76 years. The people participating in this project are diabetic patients from the San Juan de Dios Hospital in the city of Cali, Colombia, and the approval of the ethics committee of the said institution was obtained through the act CEIHSJ001-019; on the other hand, each patient signed an informed consent document so that they were aware of the procedure that was going to be performed with the electrical bioimpedance measurement equipment. Diabetic and nondiabetic patients were properly diagnosed by a doctor, with this scientifically ensuring that the study population is consistent and meets the relevant inclusion criteria. Among the participants, there were 20 people diagnosed with type II diabetes. An average of 5 impedance measurements was taken in the upper part of each person's forearm as shown in Figure 2.

The article "Noninvasive Prototype for Type 2 Diabetes Detection" was published in 2021. Journal: J Healthc Eng.

#### 2.6.2. Statistical Validation and Visualization of Principal Components

Figure 3 shows the training and prediction process based on the ATSS algorithm. Once the initial model is obtained, the training samples are added, and the performance indicators are verified to retrain the algorithm and obtain the new model.

The final population is used to obtain the model and make the predictions. For a prediction, the following procedure is done.

10 measurements are taken and the correlation verification of each of the samples is carried out with the function of

(14) $$\begin{array}{c} y=\text{a}x^{b}, \end{array}$$

where *a* is the coefficient, *b* is the exponent, the variable *x* corresponds to the frequency, and the variable *y* is the amplitude of the impedance.

The measurements are sent to the API and the model is used to predict each of the samples.

A voting process is carried out which consists of evaluating whether 80% of the predictions fall within a class, and the result is taken as a valid prediction; otherwise, it is taken as undefined (it could not be classified between diabetic or not diabetic).

p_0_ is the total coincidence probability and p_e_ is the hypothetical coincidence probability. The higher the value of the coefficient, the lower the possibility that the labels resulting from the prediction have been assigned by chance.

The process shown in Figure 4 is repeated 30 times, each time using a random order. In this way, 150 accuracy results are obtained for both the traditional method and the use of the proposed algorithm. Then, the means of the accuracies are calculated, and the Wilcoxon test is performed [22].

The article "Noninvasive Prototype for Type 2 Diabetes Detection" was published in 2021. Journal: J Healthc Eng.

Finally, the principal component analysis (PCA) is carried out, which allows reducing the dimensionality of the characteristics taken and maintaining the highest possible variance [23]; in this way, they can be reduced to only 2 dimensions and be plotted.

## 3. Results

### 3.1. BDD Prototype

Figure 4(a) shows the equipment implemented in its final form, and Figure 4(b) presents the 3d design of the housing of the bioimpedance acquisition system equipment. As can be seen in Table 3, the physical characteristics of the prototype make it possible for it to be handled with one hand in a comfortable way. The prototype delivers a prediction in 2 : 45 minutes, which is much less than waiting for laboratory analysis. On the other hand, the 9 hours of autonomy allow the prototype to be used in rural areas and 180 predictions could be made before having to charge or change the battery.  Table 4 shows the error percentages of the prototype.

Figure 5 shows that, with only 12 parts, the device can be assembled and that its implementation is simple which makes most of the cost only come from the PmodIA.

Figure 6 presents the results obtained when taking measurements of the same person during a 12-hour interval starting at 8 : 00 am and ending at 8 : 00 pm; during each hour of that interval, 10 measurements were taken.  Figure 6(a) is the bar diagram of the relative percentage of standard deviation (RSD%) that shows only a variation of 2% and this is confirmed with the graphs of Figure 6(b), where it is shown that the 120 measurements overlap.

This is an unexpected result as a person's glucose value changes throughout the day. This allows us to infer that the bioimpedance value does not depend only on glucose in the blood and that there are other factors, such as those mentioned by Punter-Villagrasa and others [24], and possibly these other parameters do remain stable during the day.

Figure 7 shows the views of the data acquisition prototype screen; the interface is intuitive in relation to its operation and the presentation of results.

To comply with the IEC 60601-1 standard, the device is designed in such a way that the battery can be removed for charging; thus, it can be ensured that the device will not be connected to the electrical network, while a measurement is taken and that these are only taken using the battery, which is why we do not have any of the leakage currents described by the standard. In addition, tests were carried out in the metrology laboratory of the Santiago de Cali University where its operating conditions were validated.

### 3.2. API Implemented

Figure 8 shows the views of the API graphical interface.  Figure 8(a) is the general database, where you can perform the data download process and system training and delete all data and input to observe the confusion matrix. Finally, Figure 8(b) shows the graph corresponding to the correlation of the amplitude dispersion data for all the frequencies defined by the acquisition system.

The article "Noninvasive Prototype for Type 2 Diabetes Detection" was published in 2021. Journal: J Healthc Eng.

### 3.3. Selection of Characteristics, Machine Learning, and Electrodes

Table 5 shows the accuracy of the learning machines using the bioimpedance characteristics. The results found show that the algorithm based on RL presents the best performances with the characteristics used.  Table 6 shows that, using biometric data, precision is increased by 7%. This is possible because there are characteristics that represent risk factors for having T2D, such as overweight and age. In addition, it has been noted that the impedance values of women are usually lower than those of men, and adding the gender tag allows the machine to assign weights more precisely. On the other hand, in the works of Nguyen et al. [25] and Chatrati et al. [26], deep learning was used to obtain accurate values above 80%; however, the use of deep learning was not implemented in BDD due to the difficulty that its implementation in a microcontroller would entail, which can be a limitation of the system and could be tested in future work.

Table 7 shows that the 3M electrodes have the lowest impedance value; therefore, they are better for this job as they add fewer impedance components. On the other hand, the classification results in Table 8 show that both the traditional method and the use of the proposed algorithm have success rates above 90%. However, the use of the active learning algorithm presents an increase in precision with a statistical significance of one (*p* < 0.05), in addition to improving the Kappa coefficient [27]; therefore, the proposed algorithm increases the predictive capacity of the system. With the improvement in precision and the Kappa coefficient that the population selection gives, it can be inferred that not all samples provide useful information and there are even some that provide information that reduces the predictive capacity of the model; this can be given because either the person, despite not having a diagnosis of diabetes, may have high impedance values or possibly have signs of prediabetes or the person has a diagnosis of diabetes but has managed the treatment of diabetes very well and managed to stop the cell damage caused by the disease.

It is important to mention that doing statistical tests is important since they allow us to establish the validity of the results regardless of which samples are used to train and validate the system in addition to showing that the results of one algorithm are greater than the other and that this relationship has significance.

The article "Noninvasive Prototype for Type 2 Diabetes Detection" was published in 2021. Journal: J Healthc Eng.

### 3.4. Classification Results

Table 8 shows the results of the performance indicators of the logistic regression machine based on traditional supervised training and with the ATSS algorithm. The mean values of accuracy were obtained with a standard deviation of 0.1313 and 0.1328 (for the algorithm without and with active learning, resp.). It also shows the *p* value results under the Wilcoxon and Kappa tests.

Figure 9 shows the results of the algorithm based on traditional training.  Figure 10(a) shows the graphical representation of the data distribution using two main components of the seed simples and Figure 10(b) shows how the adequate selection of the samples according to the SW allows the samples used by the system to present a greater separation in the classes than those found using the traditional training method.

In the literature, no works were found where the development of portable noninvasive bioimpedance equipment is presented and that also uses machine learning. Therefore, the references that were found are related to the use of bioimpedance and its relationship with glucose; these works are not focused on prediction. Regarding the proposed algorithm, only works related to machine learning techniques were found, where samples used for training and validation were selected, the proposed algorithm has a feature selection scheme for training, and as with the prediction of new samples, the algorithm can continue its learning process.

The improvements are obtained after applying the sample selection algorithm. The PCA was used to show graphically how it selects samples that are separated under the SW and how in the end they are more separated without using the algorithm since it is not possible to graph the 20 dimensions that would be obtained representing all the characteristics used. In numerical terms, the average SW without using the algorithm is 0.33, the average SW of the initial samples is 0.85 and finally, a difference is obtained between the SW with and without the algorithm of 0.2; however, the improvements are better represented with the results of the indicators obtained by the confusion matrix. The PCA was only used as a visual aid to graphically represent what the algorithm is executing.

## 4. Conclusions

The equipment developed is portable, safe, noninvasive, and with the potential to have accuracy rates above 90% that allow determining whether a person has type 2 diabetes. The active learning algorithm not only improves performance but also offers protection to the prediction model since only samples that are close to their class and that improve the performance indicators are accepted. This combined with the API allows the system to be used, retrained, and validated in different regions by different users at the same time.

The article "Noninvasive Prototype for Type 2 Diabetes Detection" was published in 2021. Journal: J Healthc Eng.

Compared to the state of the art, the BDD system does not use invasive methods or medical records of the person for prediction. In addition, it is faster than invasive tests since no laboratory analysis is required, and with the use of the API, the system can be validated externally. However, the works described in the introduction use biological markers known as the level of glucose in the blood to make the machine training, which allows a clear biological explanation of why the model works. The work proposed here does not manage to explain exactly what is the biological characteristic that allows the bioimpedance to detect diabetes, although the hypothesis of the cellular damage that the cells present is being measured with bioimpedance is presented. Therefore, this work focused on the electronic and programming design of a system capable of predicting diabetes.

All these factors and characteristics of the implemented equipment have the potential to be used in T2D screening, being a simple process; this translates into a faster diagnosis mechanism that in turn helps to reduce diseases related to T2D. This is even in health service posts in developing places where invasive diagnostic tests are difficult to access. With this development, there is a contribution to preventive medicine, which precisely meets the needs of people, in this case with type 2 diabetes. This equipment does not replace the conventional methods of detection of the pathology, but it does allow detection of this in less than 3 minutes and at any time of the day.

One of the main objectives of this research was to develop portable and low-cost equipment, so it was decided to use the ESP32 microcontroller; consequently, the development of deep learning with such hardware becomes complicated. On the other hand, with the results of above 90% accuracy, the use of a device with greater processing and memory such as a Raspberry Pi was not justifiable, which would increase the size, weight, and cost of the device in addition to reducing autonomy.

In future work, the algorithm can be modified to use sugar levels measured by noninvasive techniques such as photoplethysmography to deliver a prediction of the disease together with the glucose level.

## Figures and Tables

**Figure 1:** API's information model flow diagram.

**Figure 2:** Location of electrodes for taking measurements.

**Figure 3:** ATSS-based training and prediction process.

The article "Noninvasive Prototype for Type 2 Diabetes Detection" was published in 2021. Journal: J Healthc Eng.

**Figure 4:** Data acquisition prototype implemented. (a) Final Implementation. (b) 3d design.

**Figure 5:** Electrical diagram for the bioimpedance acquisition system.

**Figure 6:** Variation of 120 measurements taken in 12 hours. (a) Graphical boxplot of RSDs%. (b) Graphs for 120 measurements taken in a 12-hour interval.

**Figure 7:** Acquisition system views.

**Figure 8:** Views of the API's graphical interface. (a) Database. (b) Scatter plot over the entire frequency range.

**Figure 9:** Traditional training's PCA model of two main components.

**Figure 10:** ATSS′ PCA model with two main components. (a) Seed samples. (b) Samples after ATSS.

**Table 1:** System parts list.

Description	Quantity
PmodIA, programmable bioimpedance analyzer-AD5933	1
Esp32-OLED 0.96 development board with 18650 battery holder	1
1K ohm resistors	4
Two-terminal push buttons	4
4800 mAh 18650 battery	1
Adhesive electrodes	2

**Table 2:** Configuration and calibration values.

Characteristic	Value
Calibration resistance	470 Ω
Multiplier	x4
Number of cycles	511
Output voltage	2 vpp
Programmable gain	x1
Feedback resistance	20 Ω
Internal clock	Selected
Start frequency	10000 Hz
Number of steps	255
Frequency increment	280 Hz

**Table 3:** Characteristics of the acquisition equipment.

Characteristic	Value
Length	13 cm
Width	6.5 cm
High	4.0 cm
Weight	204.7 g
Autonomy with 4800 mAh battery	9 hours
Time it takes to do 10 measurements	2 : 45 minutes

**Table 4:** Percentages of equipment error.

Characteristic	Value (%)
Magnitude error	4
Phase error	4

**Table 5:** Accuracy of machines that presented the best performances.

Algorithm	Accuracy
RL with lbfgs	0.94
RL with Newton-cg	0.93
RL with liblinear	0.93
RL with sag	0.85
ANN [ 19 14 16] ^*∗*^	0.88
KNN with neighbors = 1	0.85
KNN with neighbors = 2	0.88
KNN with neighbors = 3	0.82
KNN with neighbors = 4	0.82

^*∗*^19 neurons in the input layer, 14 neurons in the hidden layer, and 16 neurons in the output layer.

**Table 6:** Statistical analysis of the selection of characteristics.

Biometric data	Model	*p* value	Significant	Accuracy
Yes	Chi-squared	1.1265*e*^−27^	Yes	0.97
Yes	Hosmer	7.6861*e*^−38^	Yes	
No	Chi-squared	2.1396*e*^−22^	Yes	0.90
No	Hosmer	1.4073*e*^−05^	Yes	

**Table 7:** Characterization of the electrodes.

Model	Average impedance value Magnitude (Ω) ∟angle [^º^]
3M	35 ∟0.03
Skintac	173 ∟0.02

**Table 8:** Performance indicators of the training model.

Indicator	Traditional training	ATSS
Accuracy	0.9300	0.9638
Kappa	0.8108	0.9171
Wilcoxon	9.1682 *e*^−20^	

## Data Availability

The data can be requested at javier.castillo00@usc.edu.co, adrian.valencia02@usc.edu.co, luis.rodriguez11@usc.edu.co, and http://www.usc.edu.co.
